# An Exosome-Related Long Non-coding RNA (lncRNA)-Based Signature for Prognosis and Therapeutic Interventions in Lung Adenocarcinoma

**DOI:** 10.7759/cureus.47574

**Published:** 2023-10-24

**Authors:** Jinghong Li, Junhua Wang, Zhihong Chen, Pan Hu, Xiaodan Zhang, Xiaojun Guo, Xiao Zhu, Yongmei Huang

**Affiliations:** 1 Computational Oncology Laboratory, Marine Biomedical Research Institute, Guangdong Medical University, Zhanjiang, CHN; 2 Oncology Department, Qingdao Hospital, University of Health and Rehabilitation Sciences (Qingdao Municipal Hospital), Qingdao, CHN; 3 Genetics Department, Marine Biomedical Research Institute, Guangdong Medical University, Zhanjiang, CHN

**Keywords:** tumor microenvironment, prognostic model, lung adenocarcinoma, exosome-related lncrna, drug therapy

## Abstract

Background

The poor prognosis of lung adenocarcinoma (LUAD) has been confirmed by a large number of studies, so it is necessary to construct a prognosis model. In addition, exosome is closely related to tumors, but there are few studies on exosome-related long non-coding RNA (lncRNA) (ExolncRNA).

Methods

In this study, we designed a prognostic model, exosome-related lncRNA-based signature (ExoLncSig), using ExolncRNA expression profiles of LUAD patients from The Cancer Genome Atlas (TCGA). ExolncRNAs were identified through univariate and multivariate and Lasso analyses. Subsequently, based on the ExoLncSig, gene ontology (GO), Kyoto Encyclopedia of Genes and Genomes (KEGG) analysis, immune function and immunotherapy analysis, drug screening, and so on were performed.

Results

AC026355.2, AC108136.1, AL590428.1, and LINC01312 were examined to establish the ExoLncSig. Gene enrichment analysis identified potential prognostic markers and therapeutic targets, including human leukocyte antigen (HLA), parainflammation, chemokine receptor (CCR), antigen-presenting cell (APC) co-inhibition, cancer-associated fibroblast (CAF), and myeloid-derived suppressor cell (MDSC). Moreover, we ascertained that the high-risk subgroup exhibits heightened susceptibility to pharmaceutical agents.

Conclusion

Our findings indicate that ExoLncSig holds promise as a valuable prognostic marker in LUAD. Furthermore, the immunogenic properties of ExolncRNAs may pave the way for the development of a therapeutic vaccine against LUAD.

## Introduction

According to global cancer statistics, lung cancer stands out as one of the most perilous malignancies [1]. Lung adenocarcinoma (LUAD), constituting approximately 40% of all lung cancer cases, represents the predominant histological subtype. Unraveling the intricacies of lung cancer pathogenesis and treatment has emerged as a focal point of research, with long non-coding RNA (lncRNA) emerging as a pivotal player in tumor initiation and progression [2].

Exosomes, nanovesicles residing within the cellular microenvironment, encompass a diverse cargo of nucleic acids, proteins, enzymes, and other biomolecules. Functioning as natural nanocarriers and intercellular messengers [3], they are released from cells through the fusion of multiple vesicles with the plasma membrane, subsequently disseminating through various biological fluids within the body. Consequently, exosomes serve as vehicles for the delivery of a myriad of bioactive substances to target cells, assuming a pivotal role in the regulation of intercellular communication [4]. Their involvement in the pathogenesis of numerous diseases, particularly cancer, is attributed to their ability to transmit genetic information [5].

In recent years, exosomes have emerged as a prominent focus in medical research, with numerous advancements made in the field of pan-cancer. Exosomes, acting as carriers of oncogenic information, play a crucial role in the pathogenesis and drug resistance of breast cancer and serve as novel markers for this disease [6]. Furthermore, exosomes are involved in the regulation of cell differentiation and tissue development, contributing to the metastasis of liver cancer, and can serve as valuable biomarkers for the clinical prediction and diagnosis of this malignancy [7]. As intercellular mediators of immune escape and tumorigenesis, exosomes play a significant role in hematological malignancies. They actively participate in the immune response of leukemia cells and have emerged as effective immunotherapeutic agents for the treatment of this disease [8].

We contend that exosome-related lncRNAs (ExolncRNAs) possess the ability to transmit immune signals that correspondingly participate in the dissemination of oncogenic information. Moreover, they regulate gene expression to govern the generation and release of exosomes, thereby orchestrating the onset of cancer. Furthermore, lncRNAs can be extracted from the surface of primitive cells in the form of exosomes, subsequently disseminating to neighboring cells or distant organs through the circulatory system, thereby facilitating tumor metastasis [9]. In this study, we aimed to develop a novel prognostic marker and explore potential immunotherapeutic targets for lung adenocarcinoma (LUAD) based on the association between exosomes, long non-coding RNAs (lncRNAs), and tumor progression.

## Materials and methods

The complete process of data analysis is drawn in Figure 1.

**Figure 1:** The flow diagram of the study process. LUAD, lung adenocarcinoma; TCGA, The Cancer Genome Atlas; GO, gene ontology; KEGG, Kyoto Encyclopedia of Genes and Genomes; ROC, receiver operating characteristic; lncRNA, non-coding RNA

Data source

In this investigation, ExolncRNAs were obtained from ExoBCD, ExoCarta, exoRBase, gene set enrichment analysis (GSEA), and GeneCards. ExoBCD is an all-encompassing repository of exosome research in breast cancer (https://exobcd.liumwei.org/) [10]. ExoCarta serves as the pioneering comprehensive database of exosome markers (http://exocarta1.latrobe.edu.au/index.html) [11]. exoRBase stands as the human blood exosome RNA database (http://www.exorbase.org/exoRBase/toIndex) [12]. By utilizing GSEA, we acquired genes from http://amigo.geneontology.org/amigo/term/GO:0000177, http://amigo.geneontology.org/amigo/term/GO:0000176, http://amigo.geneontology.org/amigo/term/GO:0071971, and http://www.wikipathways.org/instance/WP4301_r97800 [13]. GeneCards, a comprehensive database of human genes (http://www.genecards.org/), harbors 4580 exosome-related genes, from which we extracted 53 genes with a relevance score of 5 or higher. After eliminating duplicate genes, a total of 340 ExolncRNAs were procured.

Moreover, a cohort of 504 LUAD patient samples (494 tumors and 10 normal) was obtained from The Cancer Genome Atlas (TCGA). These samples contained clinicopathological characteristics, including overall survival (OS), survival status, age, gender, race, tumor (T) classification, node (N) classification, and metastasis (M) classification. Additionally, we acquired mRNA and lncRNA expression profiles of LUAD patients from TCGA.

Identification of ExolncRNAs

Initially, we employed the "limma" package in R software (R Foundation for Statistical Computing, Vienna, Austria) to extract the expression profiles of exosome-associated mRNAs based on the mRNA expression profiles of LUAD. Subsequently, we applied the filtering criteria corFilter=0.4 and pvalueFilter=0.001 to obtain the ExolncRNA expression profiles that exhibited correlation with exosome-associated mRNAs.

Construct a prognostic model with ExolncRNAs

The "survival" package was utilized to perform univariate Cox modeling, and lncRNAs exhibiting significant correlations with OS (P<0.05) were retained for further analysis. Multivariate Cox and Lasso regression analyses were subsequently employed to refine the selection of lncRNAs with regression coefficients. Then, we randomly partitioned the patients into a train set and a test set. Exosome-related lncRNA-based signature (ExoLncSig) (risk score) was calculated using the ExolncRNA expression profiles of the train set, utilizing the following formula: ExoLncSig=∑ki=1Coef(i)*ExpGene(i) (where k represents the number of ExolncRNAs, Coef denotes the regression coefficient for each ExolncRNA, and ExpGene signifies the expression level of ExolncRNA in the patient sample).

Subsequently, we calculated risk scores for patients in the train and test sets and then combined them into an all set. The median value of each set was employed as the cutoff point, dividing patients into high-risk and low-risk groups.

Survival analysis and risk curve for three sets

For survival analysis, we utilized the "survminer" and "survival" packages, which encompassed the Kaplan-Meier method and log-rank test. Subsequently, we generated risk curves and survival state curves and employed the "pheatmap" package to create a risk heatmap.

Clinical evaluation of prognostic model quality

To illustrate the relationship between clinicopathological characteristics and risk scores, we generated boxplots using the "limma" and "ggpubr" packages. Additionally, we performed univariate and multivariate independent prognostic analyses for further evaluation.

Validation of the independent prognostic model

We employed the receiver operating characteristic (ROC) curve of survival time, the clinical ROC curve [14] for one, three, and, five years, and the C-index model to evaluate the independent prognostic model.

Establishment and validation of the nomogram

Based on the aforementioned multifactorial independent prognostic model, we employed the "rmt" package to construct a nomogram capable of predicting survival over one, three, and five years. Finally, we validated the nomogram using a calibration curve.

Assessment of grouping between high and low risks

To analyze the disparity in survival between high- and low-risk groups for each clinicopathological characteristic, we employed Kaplan-Meier methods. Principal component analysis (PCA) was utilized to confirm the differentiation of high- and low-risk groups by combining mRNAs, lncRNAs, and all gene expression profiles.

Gene ontology (GO) and Kyoto Encyclopedia of Genes and Genomes (KEGG) enrichment analysis

Initially, lncRNAs that exhibited differential expression in high- and low-risk groups were filtered based on logFCfilter=1 and fdrFilter=0.05. Subsequently, we performed GO and KEGG enrichment analysis on the filtered lncRNAs. The "clusterProfiler" package was utilized for gene ontology function annotation to explore and determine their potential biological functions [15]. The resulting functional and signaling pathways associated with these lncRNAs were identified using the "GOplot" package, with "ggplot2" and "Enrichplot" packages serving as dependencies.

Differential analysis of immune function events

We downloaded 13 immune events and related genes from studies, encompassing antigen-presenting cell (APC)_co_inhibition, APC_co_stimulation, chemokine receptor (CCR), checkpoint, cytolytic_activity, human leukocyte antigen (HLA), inflammation-promoting, major histocompatibility complex (MHC)_class_I, parainflammation, T_cell_co-inhibition, T_cell_co-stimulation, type_I_interferon (IFN)_reponse, and type_II_IFN_reponse [16,17]. The "GSVA" and "GSEABase" packages were utilized to identify the immune events exhibiting differences between the high- and low-risk groups of three sets through immune-related genes.

Analysis of tumor mutation burden (TMB)

Tumor mutation burden (TMB) could serve as a vital prognostic biomarker for tumors [18]. Using TGCA somatic mutation data, we computed TMB scores and analyzed the differences in TMB across the various risk groups of three sets. Additionally, we assessed the correlation between TMB and risk scores with OS using the Kaplan-Meier method.

Examination of tumor immune evasion and immunotherapy markers

We obtained the tumor immune dysfunction and exclusion (TIDE) score file for LUAD patients from http://tide.dfci.harvard.edu, which incorporates comprehensive omics data from published immune checkpoint blockade (ICB) trials, along with biomarkers, non-immunotherapy tumor profiles, and CRISPR screens [19]. Subsequently, we analyzed the score discrepancies of the 11 immunotherapy markers between the high- and low-risk groups of three sets and employed the "GGPubR" package to visualize the results through a violin plot.

Cancer chemotherapeutic drug screening

We employed the "pRRophetic" package [20] to compute the half maximal inhibitory concentration (IC_50_) value of chemotherapeutic agents in the high- and low-risk groups of three sets, enabling the prediction and identification of drugs with therapeutic potential in varying risk scores.

Validation and response analysis of IMvigor210 immunotherapy

We utilized the "IMvigor210CoreBiologies" package to procure pertinent data from clinical trials of urothelial bladder cancer (UBC) patients [21]. Subsequently, we calculated risk scores for UBC patients based on nine ExolncRNAs identified through Lasso analysis. We then performed survival analysis to evaluate the association between risk scores and OS and confirmed the efficacy using ROC curve analysis. Furthermore, we analyzed the variation in immunotherapy responses (including complete response {CR}, partial response {PR}, stable disease {SD}, and progressive disease {PD}) among patients with UBC in the high- and low-risk groups.

Stemness index (SI) analysis in LUAD

Stemness indices (SI) serve as a measure of the resemblance between tumor cells and stem cells. We computed the mRNA stemness indices (mRNAsi) using gene expression data obtained from published literature associated with LUAD [22]. Initially, we compared the mRNAsi levels between the normal and tumor groups, followed by the Kaplan-Meier survival analysis between mRNAsi and OS. Additionally, we examined the association between mRNAsi and clinicopathological characteristics.

Statistical analysis

T-test and χ^2^ test were used to assess the difference between the two groups. P<0.05 (P<0.05; P<0.01; P<0.001) was statistically significant. Univariate and multivariate Cox analysis and Lasso analysis were used to analyze the relationship between variables and OS. The Kaplan-Meier method was used to analyze the relationship between risk score and OS. For the evaluation of accuracy, we utilized the ROC curve with the area under the curve (AUC) [23]. A higher AUC (>0.5) indicated superior modeling quality.

## Results

Analysis of patient samples

A total of 494 patient samples were randomly divided into a training set consisting of 330 samples and a test set comprising 164 samples. A comprehensive analysis of two sets revealed that the P-values of all clinicopathological characteristics exceeded 0.05 (Table 1), indicating that the differences were not statistically significant and the groups were well-defined.

**Table 1:** Clinical features of LUAD patients in the train, test, and total sets. LUA, lung adenocarcinoma; T, tumor; N, node; M, metastasis

Feature	Type	Total	Test	Train	P-value
Fustat	Alive	190 (64.63%)	52 (59.77%)	138 (66.67%)	0.3196
	Dead	104 (35.37%)	35 (40.23%)	69 (33.33%)	
Age	≤65	147 (50%)	41 (47.13%)	106 (51.21%)	0.6093
	>65	147 (50%)	46 (52.87%)	101 (48.79%)	
Gender	Female	155 (52.72%)	49 (56.32%)	106 (51.21%)	0.5005
	Male	139 (47.28%)	38 (43.68%)	101 (48.79%)	
Race	American Indian or Alaska Native	1 (0.34%)	1 (1.15%)	0 (0%)	0.1509
	Asian	5 (1.7%)	3 (3.45%)	2 (0.97%)	
	Black or African American	27 (9.18%)	6 (6.9%)	21 (10.14%)	
	White	261 (88.78%)	77 (88.51%)	184 (88.89%)	
Stage	Stage I	153 (52.04%)	41 (47.13%)	112 (54.11%)	0.4119
	Stage II	72 (24.49%)	20 (22.99%)	52 (25.12%)	
	Stage III	51 (17.35%)	19 (21.84%)	32 (15.46%)	
	Stage IV	18 (6.12%)	7 (8.05%)	11 (5.31%)	
T	T1	96 (32.65%)	30 (34.48%)	66 (31.88%)	0.9683
	T2	162 (55.1%)	46 (52.87%)	116 (56.04%)	
	T3	23 (7.82%)	7 (8.05%)	16 (7.73%)	
	T4	13 (4.42%)	4 (4.6%)	9 (4.35%)	
M	M0	276 (93.88%)	80 (91.95%)	196 (94.69%)	0.5317
	M1	18 (6.12%)	7 (8.05%)	11 (5.31%)	
N	N0	189 (64.29%)	52 (59.77%)	137 (66.18%)	
	N1	60 (20.41%)	19 (21.84%)	41 (19.81%)	
	N2	45 (15.31%)	16 (18.39%)	29 (14.01%)	

Construction of the prognostic model

A total of 281 ExolncRNAs were identified through univariate Cox analysis and further narrowed down to nine ExolncRNAs using Lasso regression analysis (Figure 2A, 2B). Subsequently, multivariate Cox analysis yielded seven ExolncRNAs along with their corresponding regression coefficients (Table 2). Only four ExolncRNAs (P<0.05) were utilized to construct an ExoLncSig. ExoLncSig=(expression level of AC026355.2)*(-0.216625)+(expression level of AC108136.1)*(0.432776)+(expression level of AL590428.1)*(0.757800)+(expression level of LINC01312)*(0.537094). Subsequently, a prognostic model was established, and patients were categorized into low-risk and high-risk subgroups based on their risk scores.

**Figure 2:** Nine ExolncRNAs selected by Lasso regression analysis and the preliminary evaluation of ExoLncSig in the train set. (A) The parameter selection of overall survival was verified by Lasso regression analysis. (B) Elucidation for Lasso coefficient profiles of nine ExolncRNAs. The risk curve (C), survival state curves(D), Kaplan-Meier survival curve (E), and risk heatmap of the seven ExolncRNAs (F) in the train set. ExolncRNAs, exosome-related long non-coding RNAs; ExoLncSig, exosome-related long non-coding RNA-based signature

**Table 2:** The regression coefficient of seven exosome-related lncRNAs. lncRNAs, long non-coding RNAs; HR, hazard ratio

Gene	Coefficient	HR	HR.95L	HR.95H	P-value
AC026355.2	-0.216625	0.805232	0.651248	0.995624	0.045450
AL691432.2	-0.226021	0.797702	0.593526	1.072114	0.134042
LINC00941	0.141132	1.151576	0.978871	1.354752	0.088686
AC108136.1	0.432776	1.541531	1.154683	2.057982	0.003330
AL590428.1	0.757800	2.133577	1.323227	3.440191	0.001877
MMP2-AS1	-0.206168	0.813696	0.656766	1.008124	0.059302
LINC01312	0.537094	1.711027	1.147474	2.551354	0.008419

Survival analysis and risk curve

In the train (Figure 2C-2F), test (Figure 3), and all (Figure 4) sets, there is a significant difference between risk score and OS in the Kaplan-Meier survival curve (P<0.05). The number of high- and low-risk groups was equal, and the proportion of deaths in the high-risk group was greater. In addition, the expressions of AC108136.1, AL590428.1, and LINC01312 were found to be elevated in the high-risk group, whereas AC026355.2 exhibited the opposite trend.

**Figure 3:** Preliminary evaluation of ExoLncSig in the test set. The Kaplan-Meier survival curve (A), risk curve (B), survival state curves (C), and risk heatmap of the seven ExolncRNAs (D) in the test set. ExoLncSig, exosome-related long non-coding RNA-based signature; ExolncRNAs, exosome-related long non-coding RNAs

**Figure 4:** Preliminary evaluation of ExoLncSig in the all set. The Kaplan-Meier survival curve (A), risk curve (B), survival state curves (C), and risk heatmap of the seven ExolncRNAs (D) in the all set. ExoLncSig, exosome-related long non-coding RNA-based signature; ExolncRNAs, exosome-related long non-coding RNAs

Clinical evaluation of the ExoLncSig

Among various clinicopathological characteristics, there was no significant difference in the risk score based on age (Figure 5A) and gender (Figure 5B). However, P<0.05 was observed in stage I versus stage II, stage I versus stage III, stage I versus stage IV, T1 versus T2, T1 versus T3, N0 versus N2, M0 versus M1 (Figure 5C-5F), while the median risk score increased with disease progression except for T4. Univariate (Figure 6A) and multivariate (Figure 6B) independent prognostic analysis revealed that the risk score (P<0.001) was significantly associated with patient prognosis. The time-dependent ROC curve demonstrated that AUC values were 0.746, 0.697, and 0.692 at one, three, and five years, respectively, indicating a high predictive accuracy (AUC>0.5) of the risk score for prognostic (Figure 7A). Notably, the clinical ROC curve and C-index curve indicated good performance for the risk score, stage, T, and N in prognosis (AUC>0.5), with the risk score exhibiting the highest AUC value (Figure 7B-7D) and concordance index (Figure 8A).

**Figure 5:** The correlation analysis between six clinicopathological characteristics and risk score. The correlation analysis for the six clinicopathological characteristics of LUAD patients, including age (A), gender (B), stage (C), tumor (T) classification (D), node (N) classification (E), and metastasis (M) classification (F). LUAD: lung adenocarcinoma

**Figure 6:** The univariate (A) and multivariate (B) independent prognostic analysis of eight clinicopathological characteristics.

**Figure 7:** Validation of the independent prognostic model. (A) The ROC curve for OS prediction includes one-, three-, and five-year LUAD patients. The ROC curve for the independent prognostic model based on eight clinicopathological characteristics includes one (B), three (C), and five (D) years. AUC, under the curve; ROC, receiver operating characteristic; OS, overall survival; LUAD, lung adenocarcinoma; T, tumor; N, node; M, metastasis

**Figure 8:** C-index curve for the independent prognostic model and the establishment and validation of a nomogram. (A) C-index curve for the clinical independent prognostic model. (B) Nomogram of the multifactorial independent prognostic model. (C) Calibration curve for the nomogram including one, three, and five years. OS, overall survival; T, tumor; N, node; MNA, metastasis not available

Function and accuracy of nomogram

The nomogram, which integrates all clinical index scores to calculate the total point, provides a comprehensive prediction of patients' survival probabilities at one, three, and five years. Risk score (P<0.001) and stage (P<0.05) exhibited significant associations with survival prediction (Figure 8B). Moreover, the calibration curve demonstrated that the curve at one, three, and five years closely approximated the true survival-predicted line, thereby validating the reliable predictive ability of the nomogram (Figure 8C).

Kaplan-Meier survival curve in clinicopathological grouping validation

The Kaplan-Meier survival curve indicated significant survival differences (P<0.05) between the high- and low-risk groups in terms of death, age (>65 and ≤65), Black or African American race, White race, gender, stages I and Ⅱ, T1-3, N0, and M0 (Figure 9A-9N).

**Figure 9:** Grouping validation of the prognostic model. The Kaplan-Meier survival analysis between risk score and OS in each clinicopathological characteristic, including dead (A), age over 65 (B), age less than or equal to 65 (C), Black or African American (D), White (E), male (F), female (G), stage I (H), stage II (I), T1 (J), T2 (K), T3 (L), N0 (M), and M0 (N). OS: overall survival

PCA of prognostic model

In Figure 10A-10C, there was a mixture of high- and low-risk groups, while in Figure 10D, the discrimination between patients in the high- and low-risk groups based on ExolncRNAs was evident.

**Figure 10:** Principal component analysis (PCA) between high- and low-risk groups. PCA in high- and low-risk groups based on mRNAs (A), lncRNAs (B), both mRNAs and lncRNAs (C), and ExolncRNAs (D). lncRNAs, non-coding RNAs; ExolncRNAs, exosome-related long non-coding RNAs

GO term and KEGG pathway involved in lncRNAs with differential expression

A total of 517 lncRNAs (P<0.05) exhibiting differential expression between patients in the high- and low-risk subgroups were identified. Subsequent GO analysis revealed that these lncRNAs are associated with the molecular function (MF) of signal receptor activation and receptor-ligand activity. In terms of biological process (BP), they are implicated in the negative regulation of proteolysis, processing, and maturation, as well as signal release and humoral immunity. Regarding cellular components (CC), they are linked to the formation of vesicle lumen, secretory granule lumen, and gap junctions (Figure 11A). Furthermore, KEGG analysis demonstrated that these lncRNAs are involved in the complement and coagulation cascade, as well as amoebiasis signaling pathways (Figure 11B). Finally, a selective listing of eight functional pathways, two signaling pathways, and the corresponding lncRNAs participating in these pathways was generated (Figure 11C, 11D).

**Figure 11:** GO and KEGG functional enrichment analysis of exosome-related genes. The GO pathways (A) and KEGG pathways (B) of 517 lncRNAs with differential expression in high- and low-risk groups. Two KEGG pathways (C) and eight GO pathways (D) with lncRNAs involved in these pathways. GO, gene ontology; KEGG, Kyoto Encyclopedia of Genes and Genomes; lncRNAs, long non-coding RNA

The investigation of immune function

The heatmap revealed that in the train set, HLA-related genes (P<0.001) exhibited low expression in the high-risk group (Figure 12A). Genes related to parainflammation, chemokine receptor (CCR), and APC co-inhibition were all highly expressed in the high-risk group (P<0.05) in the test set (Figure 12B). In the all set, HLA-related genes (P<0.001) displayed low expression in the high-risk group (Figure 12C).

**Figure 12:** Differential expression analysis of immune function based on ExoLncSig. The heatmap of the study on immune function in train (A), test (B), and all (C) sets. ExoLncSig, exosome-related long non-coding RNA-based signature; IFN, interferon; HLA, human leukocyte antigen; APC, antigen-presenting cell; CCR, chemokine receptor; MHC, major histocompatibility complex

Analysis of tumor mutation burden (TMB)

There was no statistically significant difference (P>0.05) in TMB scores between the high- and low-risk groups (Figure 13A-13C). In the train set, patients with low TMB scores and low-risk scores exhibited higher survival rates (Figure 13D), while in the test and all sets, patients with high TMB scores and low-risk scores demonstrated higher survival rates (Figure 13E, 13F).

**Figure 13:** The tumor mutation burden (TMB) analysis based on ExoLncSig. The violin plots of difference analysis in TMB between high- and low-risk score patients in the train (A), test (B), and all (C) sets. The Kaplan-Meier survival analysis of LUAD patients combined with risk scores and TMB in train (D), test (E), and all (F) sets. ExoLncSig, exosome-related non-coding RNA-based signature; LUAD, lung adenocarcinoma

Analysis of immunotherapy markers

A total of 11 immunotherapy markers, namely, TIDE, interferon gamma (IFNG), microsatellite instability (MSI), Merck18, cluster of differentiation (CD) 274, CD8, dysfunction, exclusion, MDSC, CAF, and tumor-associated macrophages M2 (TAMM2), were evaluated. Violin plots revealed that patients in the low-risk group exhibited higher scores of the TIDE, IFNG, Merck18, dysfunction, and TAMM2 in the train (Figure 14A-14E)and all sets (Figure 15A-15E). Conversely, the score of exclusion, MDSC, and CAF was higher in the high-risk group (Figure 14F-14H and Figure 15F-15H). In the test set, only the score of CAF was higher in the high-risk group (Figure 15I), while no statistically significant difference was observed between the low-risk and high-risk groups for the other markers.

**Figure 14:** Differential analysis of immunotherapy markers between high- and low-risk groups in the train set. The violin plots of TIDE (A), IFNG (B), Merck18 (C), dysfunction (D), TAMM2 (E), exclusion (F), MDSC (G), and CAF (H) in the train set. TIDE, tumor immune dysfunction and exclusion; IFNG, interferon gamma; MDSC, myeloid-derived suppressor cell; CAF, cancer-associated fibroblast; TAMM2, tumor-associated macrophages M2

**Figure 15:** Differential analysis of immunotherapy markers between high- and low-risk groups in the test and all sets. The violin plots of TIDE (A), IFNG (B), Merck18 (C), dysfunction (D), TAMM2 (E), exclusion (F), MDSC (G), and CAF (H) in the all set. (I) The violin plot of CAF in the test set. TIDE, tumor immune dysfunction and exclusion; IFNG, interferon gamma; MDSC, myeloid-derived suppressor cell; CAF, cancer-associated fibroblast; TAMM2, tumor-associated macrophages M2

Analysis of tumor chemotherapeutic drugs

The analysis revealed that patients in the high-risk subgroup generally displayed higher sensitivity to chemotherapy drugs compared to patients in the low-risk subgroup. This included cisplatin, docetaxel, gemcitabine, paclitaxel, pazopanib, sorafenib, and sunitinib, which are commonly used chemotherapy drugs. However, low-risk patients exhibited higher sensitivity to metformin. These suggest that patients with different risk scores may benefit from different chemotherapy drugs (Figure 16, Figure 17, and Figure 18).

**Figure 16:** Drug screening based on ExoLncSig in the train set. The boxplots of eight regular drugs that have differences in drug sensitivity between high- and low-risk groups in the train set, including cisplatin (A), docetaxel (B), gemcitabine (C), metformin (D), paclitaxel (E), pazopanib (F), sorafenib (G), and sunitinib (H). ExoLncSig, exosome-related long non-coding RNA-based signature; IC_50_, half maximal inhibitory concentration

**Figure 17:** Drug screening based on ExoLncSig in the test set. The boxplots of eight regular drugs that have differences in drug sensitivity between high- and low-risk groups in the test set, including cisplatin (A), docetaxel (B), gemcitabine (C), paclitaxel (D), pazopanib (E). ExoLncSig, exosome-related long non-coding RNA-based signature; IC_50_, half maximal inhibitory concentration

**Figure 18:** Drug screening based on ExoLncSig in the all set. The boxplots of eight regular drugs that have differences in drug sensitivity between high- and low-risk groups in the all set, including cisplatin (A), docetaxel (B), gemcitabine (C), metformin (D), paclitaxel (E), pazopanib (F), sorafenib (G), and sunitinib (H). ExoLncSig, exosome-related long non-coding RNA-based signature; IC_50_, half maximal inhibitory concentration

The analysis of IMvigor210 immunotherapy associated with ExoLncSig

The survival analysis of UBC patients did not reveal any statistically significant difference in survival between high- and low-risk scores (Figure 19A). However, the ROC curve demonstrated improved performance in predicting five-year survival (AUC>0.5) (Figure 19B). Furthermore, there was no statistically significant difference (P>0.05) in response to IMvigor210 immunotherapy between high- and low-risk patients (Figure 19C).

**Figure 19:** The verification of ExoLncSig associated with IMvigor210 immunotherapy clinical trial and the mRNAsi analysis of LUAD patients. (A) The Kaplan-Meier survival analysis between risk score and OS in UBC based on ExoLncSig. (B) ROC curve to evaluate the predictive accuracy of the Kaplan-Meier survival curve mentioned above. (C) The difference of immunotherapeutic response in high- and low-risk groups in UBC. (D)The difference analysis of mRNAsi in normal and tumor sets. (E) The Kaplan-Meier survival analysis between mRNAsi and OS. The correlation analysis between mRNAsi and clinicopathological characteristics included M (F), gender (G), stage (H), and T (I). ExoLncSig, exosome-related long non-coding RNA-based signature; OS, overall survival; UBC, urothelial bladder cancer; ROC, receiver operating characteristic; M, metastasis; T, tumor; AUC, area under the curve; mRNAsi, mRNA stemness indices; CR, complete response; PR, partial response; SD, stable disease; PD, progressive disease

The mRNA stemness index (mRNAsi) analysis of LUAD

A statistically significant distinction in mRNAsi was observed between the tumor and normal groups (Figure 19D), albeit no statistically significant difference was detected in the survival of LUAD patients between those with high and low mRNAsi (Figure 19E). Correlation analysis between mRNAsi and clinicopathological characteristics revealed that patients with M1 had higher mRNAsi compared to those with M0 (Figure 19F). Males exhibited higher mRNAsi than females (Figure 19G). Additionally, mRNAsi displayed an increasing trend from stage I to stage IV, with a slight decrease in stage III (Figure 19H). Furthermore, mRNAsi increased from T1 to T3, but mRNAsi corresponding to T4 was lower than that of T2 (Figure 19I).

## Discussion

Due to the unfavorable prognosis and high incidence of LUAD, it is imperative to develop a novel prognostic model. Investigating at the genetic level can mitigate the error arising from variations in the clinical presentation of patients. Consequently, upon discovering the pivotal role of exosomes in tumor occurrence and progression, we endeavored to construct ExoLncSig to explore the potential of ExolncRNAs in predicting the survival time of LUAD.

Based on ExoLncSig with four ExolncRNAs, we deduced that AC108136.1, AL590428.1, and LINC01312 exhibited a positive correlation with patients' prognostic risk scores, signifying their status as risk genes. Conversely, AC026355.2 plays a role as a protective gene. The Kaplan-Meier survival analysis, independent prognostic analysis, and nomogram demonstrated a statistically significant association between the risk score and OS. The validation of clinicopathological groups revealed that ExoLncSig exhibited a statistically significant prognostic capability concerning age, Black or African American ethnicity, White race, gender, stages I and II, T1-3, N0, and M0. This indicates that ExoLncSig is well-suited for prognosticating early-stage LUAD.

In GO and KEGG enrichment analysis, lncRNAs are implicated in the modulation of signal receptor activation and receptor-ligand activity, as well as the negative regulation of protein hydrolysis, processing, maturation, signal release, and humoral immunity. They are also involved in functional pathways such as vesicle lumen, secretory granulosa lumen, and gap junction formation, along with the complement and coagulation cascade and amoebiasis signaling pathways. It suggests that the occurrence and development mechanism of LUAD may be associated with these pathways, and they may also serve as potential targets for treatment and prognosis.

The tumor microenvironment (TME) exerts a significant influence on tumor progression and metastasis. Our findings demonstrate the high expression of HLA in low-risk patients, supporting the notion that HLA can serve as a prognostic indicator for LUAD and a marker for anti-tumor immunity research. Furthermore, parainflammation emerges as a novel biomarker for tumors. The identification of an inflammatory response in a patient's tumor sample may facilitate the development of an anti-inflammatory-based anti-tumor regimen for individuals exhibiting a highly reactive parainflammation response [24]. Our findings indicate that genes associated with parainflammation are significantly upregulated in high-risk patients, underscoring the relevance of these genes in the treatment of LUAD. Additionally, we observed the elevated expression of genes linked to chemokine receptor (CCR) and APC co-inhibition in high-risk patients. Chemokine and chemokine receptor-based prognostic signatures have been established as reliable biomarkers for LUAD, serving as prognostic indicators for immunotherapy response [25].

Inhibiting the expression of antigen-presenting cell (APC) co-stimulatory signals weakens the anti-tumor immune response. Therefore, APC co-inhibition can serve as an indicator of prognosis in LUAD. Recent research has demonstrated that cancer-associated fibroblasts (CAFs) play a critical role in the formation and development of TME and have the potential as therapeutic targets [26,27]. In our study, we observed high expression levels of CAFs and myeloid-derived suppressor cells (MDSCs) in high-risk patients. In our perspective, inhibiting the secretion function of CAFs and their remodeling effect on the extracellular matrix of tumor cells may represent a viable approach for treating LUAD. Finally, MDSCs can downregulate T-cell receptor expression and suppress T-cell activation, thereby impairing the body's anti-tumor immune response and facilitating tumor development. Combining existing immunotherapy with MDSC inhibition has demonstrated promising outcomes and favorable tolerability in cancer treatment [28].

Patients with different risk scores exhibit varying sensitivities to chemotherapy drugs. The ExoLncSig can aid in the identification of suitable chemotherapy drugs and improve prognostic outcomes. Our data analysis unveiled a significant elevation in mRNAsi within the tumor group; however, there was no significant correlation between mRNAsi and risk score. The inexhaustible proliferative attributes of cancer stem cells have a direct impact on the resistance to LUAD therapies. Analyzing the mRNAsi aids in formulating tailored treatment strategies for patients. Moreover, impeding the distinctive features of cancer stem cells has emerged as a promising avenue for identifying novel targets in LUAD treatment [29].

The association between ExoLncSig and the tumor immune microenvironment aligns with the findings of the recent investigation. Nonetheless, our study does have certain limitations. Firstly, the modeling was based on a small number of patient samples solely obtained from TCGA. Secondly, ExoLncSig could not be applied in TMB analysis or IMvigor210 immunotherapy analysis.

Additionally, RNA vaccines have emerged as a novel modality in tumor immunotherapy. Li et al. have discovered an immunogenic long non-coding RNA, namely, LIMIT, which augments the expression of MHC-Ⅰ in tumor cells among melanoma patients [30]. We believe that further investigations into the immunogenicity of ExolncRNAs and the associated signaling pathways could pave the way for the development of therapeutic vaccines or targets specific to LUAD.

In general, ExolncRNAs possess considerable potential as prognostic indicators for LUAD. Moreover, ExoLncSig enables the computation of patients' risk scores, facilitating the identification of immunotherapy targets and medications based on these scores.

## Conclusions

In summary, we have developed ExoLncSig, a composite of four ExolncRNAs, namely, AC026355.2, AC108136.1, AL590428.1, and LINC01312. As a novel prognostic marker, it enables the prediction of survival rates in LUAD patients, analysis of the tumor immune microenvironment status, immunotherapy, and drug screening.
